The article "Leadership empowering behaviour as a predictor of employees’ psychological well-being: Evidence from a cross-sectional study among secondary school teachers in Kohat Division, Pakistan" was retracted in 2025. Reasons: lack of ethics approval or compliance; missing or withdrawn patient consent; concerns about the welfare of human subjects.

# Leadership empowering behaviour as a predictor of employees’ psychological well-being: Evidence from a cross-sectional study among secondary school teachers in Kohat Division, Pakistan

**DOI:** 10.1371/journal.pone.0254576

**Published:** 2021-07-22

**Authors:** Qaiser Suleman, Makhdoom Ali Syed, Saqib Shehzad, Ishtiaq Hussain, Alam Zeb Khattak, Irfan Ullah Khan, Muhammad Amjid, Iqleem Khan

**Affiliations:** 1 Elementary & Secondary Education Department, Government of Khyber Pakhtunkhwa, Peshawar, Pakistan; 2 Department of Education, University of Kotli, Kotli, Azad Jammu & Kashmir, Pakistan; 3 Department of Education, Abdul Wali Khan University Mardan, Mardan, Pakistan; 4 Department of Education & Psychology, Kohat University of Science & Technology, Kohat, Pakistan; 5 Department of Psychology, International Islamic University, Islamabad, Pakistan; 6 Department of Education & Research, University of Lakki Marwat, Lakki Marwat, Pakistan; Uniwersytet Slaski w Katowicach, POLAND

## Abstract

In this technologically developed scenario, many organizations in developing countries including Pakistan have expanded the enthusiasm for understanding and creating an encouraging administrative and managerial environment. Numerous organizations are struggling for structural changes by deserting the old-fashioned organizational management style and implementing an empowering leadership where leaders give more authority to subordinates in decision making and responsibilities with the aim to increase organizational productivity. Therefore, the study examined the leadership empowering behaviour as a predictor of employees’ psychological well-being of the educational institutions at secondary level in Kohat Division, Pakistan. A total sample of 564 secondary school teachers (male *n* = 379; female *n* = 185) was carefully chosen through a stratified random sampling technique. In this study, a non-experimental predictive correlational design was adopted. In order to collect data from the participants, two different standardized research tools i.e., the Leader Empowering Behaviour Questionnaire and Ryff’s Psychological Well-being Scale were used. After the collection of data, it was analyzed on the basis of mean, standard deviation, Pearson’s product-moment correlation, and multiple linear regression model. In conclusion, the study confirmed a significant positive correlation between leadership empowering behaviour and employees’ psychological well-being. Leadership empowering behaviours predict employees’ psychological well-being positively. Therefore, it was recommended that empowering behaviour might be adopted by the school leaders to improve the employees’ psychological well-being for better organizational productivity.

The article "Leadership empowering behaviour as a predictor of employees’ psychological well-being: Evidence from a cross-sectional study among secondary school teachers in Kohat Division, Pakistan" was retracted in 2025. Reasons: lack of ethics approval or compliance; missing or withdrawn patient consent; concerns about the welfare of human subjects.

## Introduction

In this technologically developed scenario, many organizations in developing countries including Pakistan have expanded the enthusiasm for understanding and creating a conducive administrative and managerial environment. Numerous organizations are striving to undergo structural changes by deserting the traditional organizational management styles and introducing an empowering leadership where leaders assign more authority in decision-making and responsibilities for subordinates’ jobs with the aim to increase organizational productivity [1]. Nowadays, organizations require workforces who are emotionally associated with their work and accept every challenge for organizational prosperity and betterment. Leaders believe that fulfilled, proficient, dedicated, and devoted employees are the most crucial asset of an organization therefore they are striving to enhance their well-being and employment. Thus, organizations regardless of scope and market, endeavor to hold the competent and best employees recognizing their significant role and impact on organizational efficiency and productivity. In order to overcome these organizational challenges, organizations ought to make potential and encouraging relationships with their employees and ensure their job satisfaction [2, 3]. Accordingly, positive psychology is considered the most important subject in the field of leadership and organizational advancement [4, 5]. Recently, researchers started to streamline the possible advantages of positive psychology in the working environment to improve organizational performance and employees’ work experience [6]. Positive psychology is a systematic and logical approach to deal with considering human feelings, thinking, sentiments, views, and behaviour, with an emphasis on qualities rather than shortcomings, constructing the decent qualities in life rather than patching the bad [7]. Positive organizational psychology tries to recognize inspirations, empowering influences, and impacts of the positive organizational approaches, know how they are stimulated, encouraged, and why they work in the first place, all in the endeavor to discover approaches to invest in their lives. This new approach increases an outstandingly positive phenomenon in numerous organizations leading towards the advancement of employees’ strong-points, boosts resilience and carries recuperating, revitalizing, and remedial capacity to the workplace [5] In a workplace, the perceptions of positive psychology are comprised of Positive Organizational Scholarship and Positive Organizational Behavior and contain domains i.e., leadership, well-being, empowerment, commitment, and engagement [8].

The article "Leadership empowering behaviour as a predictor of employees’ psychological well-being: Evidence from a cross-sectional study among secondary school teachers in Kohat Division, Pakistan" was retracted in 2025. Reasons: lack of ethics approval or compliance; missing or withdrawn patient consent; concerns about the welfare of human subjects.

Empowerment has gained the attention of researchers during the last three decades and the literature abounds with its definitions, methods of employing in the organizations, and its measurement [9]. Empowerment infers conceding essential power and self-sufficiency which empowers workers to make organizational decisions [10]. It involves supervisors to convey information and knowledge to improve employees’ work efficiency [11]. Empowering leaders authorize and inspire their workforces to regulate their work activities [12]. Hence, empowerment is exercised by the leaders to ensure employees’ advancement chances to build up skills of self-leadership, which could aid the positive reactions to new jobs and duties [13]. Menon [14] classifies empowerment into three approaches such as psychological empowerment, structural empowerment, and leadership empowerment. A leader empowering approach can be characterized as an advantageous and facilitative process where subordinates observe their leaders to ensure employees’ self-regulation, self-control, self-management, and self-leadership [15, 16].

Research has confirmed that leaders who stimulate creative-thinking energize the manifestation of numerous optimistic individuals and organizational productivity [17], which consequently develops a culture of performance and thus contributes to growing enthusiasm in understanding, envisaging, foreseeing, and promoting empowerment and empowering leadership in practice and research [13]. The idea of empowering leadership was initially developed by Manz and Sims in 1990s and they called empowering leadership as “Super Leadership” [18]. Previous research studies have revealed that leadership empowering behaviour has different sorts of work outcomes [19, 20]. Conger and Kanungo [1] expressed that empowering leadership behaviour is practiced as it enhances organizational efficiency by creating more malleability and adjustability in management and reinforcing workers’ convictions in their self-effectuality and self-efficacy and thus lessens their sense of powerlessness. It is viewed as an empowering process instead of a delegating process and is defined as the leaders’ capability to delegate authority, promote self-directed decision-making, accountability, developing skills, and training of subordinates [21, 22].

Leader empowering behaviour emphasizes the process of subordinate’s self-influence rather than level control which is completely different from the traditional style of leadership [23]. Empowering leaders will delegate responsibility, share information, boost accountability, allow participative decision-making, act as a coach, and show their concerns by listening and attending to subordinates [24]. Leadership empowering behaviour is a six-dimensional construct including delegation of authority; accountability; information sharing; skill development; self-directed decision-making; and coaching for innovative performance [22]. In the *delegation of authority*, the empowering leaders delegate authority to their subordinates to empower them so that they may play their contributory role towards effective decisions for the prosperity of the organization [21]. *Accountability for outcomes* refers to the leaders re-allocating authority as well as assigning new tasks to subordinates, making them responsible for outcomes [22]. *Information sharing* is described that leaders share information with their subordinates and the subordinates also share information with others for the smooth running of the organization [22, 25]. *Self-directed decision-making* means allowing and involving employees to take an interest in the problem-solving process making them more empowered [8, 22, 26]. In *skills development* and *coaching for innovative performance*, the leaders provide training opportunities for their subordinates to enhance their skills [22, 25].

The article "Leadership empowering behaviour as a predictor of employees’ psychological well-being: Evidence from a cross-sectional study among secondary school teachers in Kohat Division, Pakistan" was retracted in 2025. Reasons: lack of ethics approval or compliance; missing or withdrawn patient consent; concerns about the welfare of human subjects.

Due to expanding worldwide competitiveness and innovative progression in the 21st century, numerous organizations are making an effort to go through basic changes by discarding the traditional organizational approaches and adopting innovative approaches. In this regard, the idea of employees’ psychological well-being is very crucial to be considered because it causes positive organizational outcomes as well as in their personal lives. Therefore, extensive research on this subject is getting interest increasingly in the management area [27]. Actively engaged subordinates in their job can feel satisfied and inspired contributing to positive feelings of well-being [28]. Research reveals that higher psychological well-being is associated with higher employees’ efficiency and profitability [29]. The role of psychological well-being is more conspicuous in producing instead of predicting variance in performance. Employees possessing higher well-being are more committed, resilient, optimistic, and have the capability to handle the issues effectively. A significant level of psychological well-being is strongly related to various positive outcomes with respect to a professional career as well as personal life [30].

Employee psychological well-being is a multi-dimensional concept described in different ways by researchers. According to Wright [31], psychological well-being is a subjective and overall judgment that one is experiencing a maximal positive and usually minimal negative and undesirable feelings. It is the ability of an individual to feel pleased and performs successfully despite undesirable feelings which are typically the part of life [32]. Panaccio and Vandenberghe [33] defined psychological well-being as the presence of a positive effect, the absence of undesirable effect, and the joint presence of employment and life gratification. It is the individual’s assessment or appraisal of his life–either with respect to life satisfaction (intellectual appraisal) or impact (emotional reactions) which is also classified into pleasant impact (positive feelings) and horrendous impact (negative feelings) [34]. It is the individuals’ gratification—feeling better and living securely and healthily. It is comprised of all the short and long terms psychological functioning and positive well-being (e.g. positive effect, morale, and self-confidence) and negative well-being (e.g. unhappiness, discontent, discouragement, and anxiety) [35]. As per Diener and Suh [36], psychological well-being may show up in the form of thoughts or influences which is consistent with Ryff and their partners’ model of psychological well-being including six domains i.e., self-acceptance, personal growth, purpose in life, environmental mastery, positive relations with others, and autonomy [37, 38].

The article "Leadership empowering behaviour as a predictor of employees’ psychological well-being: Evidence from a cross-sectional study among secondary school teachers in Kohat Division, Pakistan" was retracted in 2025. Reasons: lack of ethics approval or compliance; missing or withdrawn patient consent; concerns about the welfare of human subjects.

Organizational efficiency and productivity depend on the employees’ fulfillment, pleasure, and good well-being [27]. Psychological well-being deals with an individual’s feeling in normal life and these feelings may be positive i.e., happiness, gratification, etc and negative i.e., dissatisfaction and depression [39]. Organizations possessing employees with strong psychological well-being are accomplishing gainful results and even employees having good psychological well-being are eager to come to work. On the other hand, employees possessing poor psychological well-being will tend to exhibit absenteeism. Individuals have respect for their colleagues provided they are participated in the decision-making process, have autonomy in working, and feel free from workload pressure. Employees desire to be sheltered, important, and fulfilled in their workplace [40]. Improving the psychological well-being of employees contributes to personal as well as organizational benefits and is the basic component of overall well-being relating to psychological well-being, longer lives, and greater happiness for employees [41]. Employees’ physical, psychological, and personal well-being may influence their productivity and efficiency. Psychological well-being is the fundamental measure of a healthy and happy life. Mentally disturbed employees will show undesirable and bothersome behaviours at work and in personal life leading to occupational stress and cause unsatisfactory performance. Long-term and extravagant stress causes a serious threat to employees’ well-being [42]. Cartwright and Cooper [43] claimed that individuals with strong psychological well-being at work are more advantageous, healthier, have more joyful lives, and live longer. Similarly, Wright and Cropanzano [44] found a positive linkage between psychological well-being and work performance.

The article "Leadership empowering behaviour as a predictor of employees’ psychological well-being: Evidence from a cross-sectional study among secondary school teachers in Kohat Division, Pakistan" was retracted in 2025. Reasons: lack of ethics approval or compliance; missing or withdrawn patient consent; concerns about the welfare of human subjects.

Previous research studies reveal extensive evidence that there is positive relationship between leadership empowering behaviour and numerous organizational outcomes such as employees’ empowerment [15, 20, 26, 45–48], work engagement [4, 49–52], task performance [12, 16, 19, 53], employees outcomes [17, 54], turnover intention [45–47, 50, 55], employees’ commitment [22, 56], customer satisfaction [57], organizational citizenship behaviours [46, 58, 59], psychological empowerment [17], employees’ commitment to organizational change [60], team performance and knowledge sharing [12], innovation [61], in-role behavior and extra-role behavior [20], creativity [9, 62], task proficiency and proactive behavior [63], job satisfaction [9, 16, 22, 56], psychological well-being [4], and subjective well-being [53]. Moreover, Suar, Tewari, and Chaturbedi [64] expressed that the successful running of an organization depends upon effective leadership that can influence organizational procedures and goals as well as employees’ beliefs, attitudes, and behaviours. Additionally, a positive approach to leadership can influence miscellaneous strengths and abilities and promote individual as well as organizational growth and development [65]. Besides, research proposes that empowering employees will bring about the experience of positive occupational cognitions, which could bring about enhanced employees’ satisfaction, performance, devotion, and willingness to remain with the organization [52, 55, 66, 67].

In the current dynamic working environment, organizations must facilitate employees and utilize them to maintain quality and competitiveness. Therefore, it is imperative to recognize the role of employees’ perceptions of their leadership contributing to the creation of a conducive working environment where they feel secure, satisfied, empowered, willing to perform effectively more than leaders’ expectations, and wish to remain in the organization [46]. In such an environment, employees’ psychological well-being is very crucial as it contributes to positive outcomes, improved work performance, and higher productivity [29, 44, 68–73]. Therefore, research is becoming more and more critical on this subject in the management and other fields [27]. Research revealed that leadership behaviour plays a very important role in enhancing employees’ job satisfaction, work motivation, well-being, and work behaviour [74–76]. On the other hand, modern organizations are increasingly conscious of the importance to sustain and promote employees’ well-being to gain and maintain competitive advantage [77]. Employees are considered the most important organizational assets which can play their role in achieving organizational goals and their performance is an important foundation stone for an organization that ensures high-quality performance thus increase organizational productivity. Research shows that employees’ psychological well-being has a positive influence on job performance [70]. Therefore, leadership and employees’ psychological well-being are two important variables to be considered in the workplace. Although there is an extensive body of literature on leadership and employees’ psychological well-being, but there is a lack of empirical research that has clearly examined the impact of leadership empowering behaviours on employees’ psychological well-being. Unfortunately, literature revealed that in Pakistan, research on leadership empowering behaviour and employees’ psychological well-being has been badly ignored although these variables in an organization are so important to be considered. Similarly, Globally, only few studies have been conducted such as Park et al. [4] who conducted a study to examine the influence of empowering leadership on the employees’ psychological well-being. So, to fill this gap in the Pakistani context, the aim of our paper is to examine leadership empowering behaviour as a predictor of employees’ psychological well-being in the workplace. The findings of the study will bring constructive revolution in organizational leadership which will play a contributory role in achieving organizational goals through psychologically healthier employees.

The article "Leadership empowering behaviour as a predictor of employees’ psychological well-being: Evidence from a cross-sectional study among secondary school teachers in Kohat Division, Pakistan" was retracted in 2025. Reasons: lack of ethics approval or compliance; missing or withdrawn patient consent; concerns about the welfare of human subjects.

## Objectives of the study

The study was aimed to examine the leadership empowering behaviour as a predictor of employees’ psychological well-being of the educational institutions at secondary level in Khyber Pakhtunkhwa, Pakistan. Therefore, the study was conducted:

1. to find out the relationship between leadership empowering behaviour and teachers’ psychological well-being at secondary level
2. to examine the leadership empowering behaviour as a predictor of teachers’ psychological well-being at secondary level.

## Research hypotheses

Hypothesis 1. *A statistically significant relationship exists between leadership empowering behaviour and teachers’ psychological well-being at secondary level*.

Hypothesis 2. *Leadership empowering behaviour positively predicts teachers’ psychological well-being at secondary level*.

## Conceptual framework of the study

A conceptual framework is the researchers’ understanding that how the variables under investigation are related to each other. It presents a plan for the research study to be followed. In more simple words, it describes scientifically and logically the actions required to be taken during the research study through a pictorial display. In this cross-sectional study, a conceptual framework has been designed regarding the leadership empowering behaviour as a predictor of employees’ psychological well-being (see Fig 1).

**Fig 1:** Conceptual framework. Indicating the Multiple Linear Regression Model between leadership empowering behaviour (independent variable) and teachers’ psychological well-being (dependent variable).

## Materials and methods

### Population

This investigation was carried out in Kohat Division located in the province of Khyber Pakhtunkhwa (Pakistan) including five districts i.e., Karak, Kohat, Hangu, Kurram, and Orakzai. In research, it is essential to present a precise population in terms of subjects or elements being investigating i.e., objects, people, association, etc. In this cross-sectional investigation, all the secondary school teachers (SSTs) in the Kohat Division were the study population. According to the Annual Statistical Report of public sector schools in Khyber Pakhtunkhwa, there were total 1882 working SSTs (Male *n* = 1261; Female *n* = 621) in government secondary schools of Kohat Division. The SSTs have been categorized in four groups i.e., SSTs (General) (Male *n* = 691; Female *n* = 397), SSTs (Information Technology) (Male *n* = 36; Female *n* = 29), SSTs (Biology/Chemistry) (Male *n* = 274; Female *n* = 110), and SSTs (Physics/Mathematics) (Male *n* = 260; Female *n* = 85) (see Table 1) [78].

**Table 1:** Study population and sample size.

Districts	SSTs (General)				SSTs (Information Technology)				SSTs (Biology/Chemistry)				SSTs (Physics/Maths)			
	Male		Female		Male		Female		Male		Female		Male		Female	
	*N*	*n*	*N*	*n*	*N*	*n*	*N*	*n*	*N*	*n*	*N*	*n*	*N*	*n*	*N*	*n*
Karak	192	58	128	38	16	05	11	03	91	27	40	12	98	29	44	13
Kohat	283	85	178	53	13	04	16	05	95	29	47	14	87	26	35	11
Hangu	105	32	46	14	06	02	01	00	41	12	13	04	34	10	04	01
Kurram	65	20	29	09	01	00	01	00	33	10	04	01	31	09	01	00
Orakzai	46	14	16	05	00	00	00	00	14	04	06	02	10	03	01	00
**Total**	**691**	**209**	**397**	**119**	**36**	**11**	**29**	**08**	**274**	**82**	**110**	**33**	**260**	**77**	**85**	**25**

**Key:** SSTs = Secondary School Teachers; *N* = Population Size; *n* = Sample Size.

The article "Leadership empowering behaviour as a predictor of employees’ psychological well-being: Evidence from a cross-sectional study among secondary school teachers in Kohat Division, Pakistan" was retracted in 2025. Reasons: lack of ethics approval or compliance; missing or withdrawn patient consent; concerns about the welfare of human subjects.

### Sample size and sampling procedure

In research, a proper determination of the sample size is a crucial phase in the design of a study. So, the validation and authentication of research findings dependent upon the appropriate sample size. According to Gay and Diehl [79], if the population size is around 1500 then 20% sample size should be selected. In this cross-sectional study, the total population size comprised 1882 participants (Male *n* = 1261; Female *n* = 621). The sample subjects were selected at the rate of 30% instead of 20% from each district to ensure valid and authentic research outcomes. In this way, a total sample of 564 SSTs (Male *n* = 379; Female *n* = 185) was carefully chosen through stratified random sampling technique including 328 SSTs (General) (Male *n* = 209; Female *n* = 119), 19 SSTs (Information Technology) (Male *n* = 11; Female *n* = 8), 115 SSTs (Biology/Chemistry) (Male *n* = 82; Female *n* = 33), and 102 SSTs (Physics/Mathematics) (Male *n* = 77; Female *n* = 25) (see Table 1).

### Research design

The research design describes the overall planning or approach that a researcher chooses to coordinate the various components of the study systematically and logically to ensure the successful resolution of the research problem [80]. In this cross-sectional study, leadership empowering behaviour was examined as a predictor of teachers’ psychological well-being and therefore, a non-experimental predictive correlational survey-based research design was applied [81]. In predictive correlational research studies, a variance of one or multiple variables is predicted on the basis of the variance of another variable(s). As with experimental designs, the study variables are categorized as independent (predictor) and dependent (outcome). So, in this study, leadership empowering behaviour is the independent variable (predictor) while teachers’ psychological well-being is the dependent variable (outcome).

### Measurements

#### Leader Empowering Behaviour Questionnaire (LEBQ)

The LEBQ constructed by Konczak, Stelly, and Trusty [22] was utilized to gauge the teachers’ perceptions of their leaders empowering behaviours. The instrument comprises of total nineteen items designed on a seven-point Likert scale i.e., 1 = Strongly Disagree; 2 = Disagree; 3 = Somewhat Disagree; 4 = Neither Agree nor Disagree; 5 = Somewhat Agree; 6 = Agree; and 7 = Strongly Agree. The instrument measures six subdomains of leadership empowering behaviours i.e., delegation of authority, self-directed decision-making, accountability for outcomes, information sharing, skills development, and coaching for innovative performance. All the subdomains of the leader empowering behaviour scale consist of three items except information sharing which has four items. The original instrument was consisted of 17 items but Bester, Stander, and Van Zyl [46] added two items on information sharing from Arnold, Arad, Rhoades, and Drasgow [24] to make it more precise. These items are: “*My manager explains his or her decisions and actions to my workgroup*” and “*My manager shares organizational goals to my workgroup*”. Konczak, Stelly, and Trusty [22] confirmed that six-factor constructs provide precise and comprehensive feedback to leadership and explain a greater percentage of the total variance. They calculated the reliability coefficients of the LEBQ as ranging between 0.82 and 0.88.

The article "Leadership empowering behaviour as a predictor of employees’ psychological well-being: Evidence from a cross-sectional study among secondary school teachers in Kohat Division, Pakistan" was retracted in 2025. Reasons: lack of ethics approval or compliance; missing or withdrawn patient consent; concerns about the welfare of human subjects.

#### Ryff’s psychological well-being scale

In order to quantify the participants’ psychological well-being, Psychological Well-being Scale (PWB) developed by Ryff [37] was utilized comprising 42 items and six subdomains i.e., autonomy, environmental mastery, personal growth, positive relations with others, the purpose of life, and self-acceptance, [37, 38]. Every subdomain is comprised of seven items designed on a 6-point Likert scale ranging from 1 = strongly disagree to 6 = strongly agree. Among these 42 items, 20 items were positively worded and scored as 6 = strongly agree to 1 = strongly disagree and the rest of the items were scored reversed because of their negative nature. The higher scores show more significant experience of psychological well-being and positive effects. Pethtel, Moist, and Baker [82] calculated satisfactory reliability for Ryff’s Psychological Well-being Scale including environmental mastery (*r* = 0.77), autonomy (*r* = 0.76), positive relations (*r* = 0.82), personal growth (*r* = 0.78), self-acceptance (*r* = 0.84), and purpose of life (*r* = 0.72). Likewise, Henn, Hill, and Jorgensen [83] also indorsed the reliability of the scale ranging from 0.86 to 0.93.

### Data collection and statistical analysis

In this cross-sectional study, the standards of research ethics were ensured to protect the subjects of its possible consequences. So, this study was reviewed and approved by the Graduate Research Committee (GRC) of the Department of Education, University of Kotli, Kotli, Azad Jammu & Kashmir. Before the commencement of the data collection process, participants were explained the facts, implications, and consequences of this study and thus obtained their informed written consent. Both the questionnaires were available in English language and distributed among the participants in the same language. Each questionnaire was comprised of a covering letter in which the research subjects were informed that filling the questionnaires would be their informed written consent for participation in this investigation. They were also provided assistance in understanding the questionnaires with respect to language. Furthermore, they were told that their responses would be destroyed after statistical analysis. Then the data collection process was initiated on February 15, 2019 and completed on November 10, 2019 successfully with 92.20% response rate (see Table 2). The researchers personally met the respondents for collecting data regarding leadership empowering behaviour and their own psychological well-being. Thus, after the completion of the data collection process, the raw data scores were accurately and properly well-ordered and presented in tables. Statistical analysis was done through Statistical Package for Social Science (SPSS) version 25.

The article "Leadership empowering behaviour as a predictor of employees’ psychological well-being: Evidence from a cross-sectional study among secondary school teachers in Kohat Division, Pakistan" was retracted in 2025. Reasons: lack of ethics approval or compliance; missing or withdrawn patient consent; concerns about the welfare of human subjects.

**Table 2:** Detail of participants’ response rate.

Gender	Questionnaires Distributed	Questionnaires Received	Response Rate in %
**Male SSTs**	379	353	93.14
**Female SSTs**	185	167	90.27
**Total**	564	520	92.20

In order to measure the leadership empowering behaviours and teachers’ psychological well-being, descriptive statistics i.e., mean, standard deviation, range, skewness, and kurtosis were applied. In order to find out the relationship between leadership empowering behaviour and teachers’ psychological well-being, Pearson’s product-moment correlation was applied to test the research hypothesis. Pearson’s correlation is a statistical test used for measuring a statistical relationship between two continuous variables. It is considered an excellent procedure for estimating the relationship between variables due to its method of covariance. It provides information about the degree of the correlation, or association, and its direction. The correlation strength was measured as 0.01≤ r ≤ 0.39 = weak relationship; 0.40 ≤ r ≤ 0.69 = moderate relationship; and r ≥ 0.70 = strong relationship [84]. To examine the role of leadership empowering behaviour as a predictor of teachers’ psychological well-being, multiple linear regression modeling (enter method) was run to explore the role of each subdimension of leadership empowering behaviour as predictor of teachers’ psychological well-being. Multiple linear regression modeling is used to measure the relationship between one continuous dependent variable and two or more independent variables. The independent variables might be categorical or continuous. So, in this study, the leadership empowering behaviour was independent variable while teachers’ psychological well-being was dependent variable.

## Results

### Participants’ demographic characteristics

In this cross-sectional investigation, 520 out of 564 secondary school teachers participated willingly at the request of the principal investigator through seeking formal permission and informed consent. In this study, only eleven demographic characteristics were studied such as gender, marital status, age, experience, nature of the job, mode of appointment, income level, academic qualification, professional qualification, and locality. To analyze the demographic characteristics of the participants, a simple percentage was used. Table 3 indicates that 344(67.88%) of the participants were males and 167(32.12%) were females. In case of marital status, 443(85.19%) participants were found married while only 77(14.81%) were found single. With respect to age, 64(12.31%) participants were in the age group 25–30 years, 128(24.62%) were in the age group 31–35 years, 113(21.73%) were in the age group 36–40 years, 132(25.38%) were in the age group 41–45 years, and 83(15.96%) were in the age group 46 years and above. In terms of experience, 119(22.88%) of participants had 1–4 years, 221(42.50%) had 5–9 years, 113(21.73%) had 10–14 years, and 67(12.88%) had 15 or more years of experience. All the participants 520(100.0%) have a regular and permanent job. In case of the mode of appointment, 141(27.12%) participants were appointed through KPPSC, 171(32.88%) were appointed through Departmental Selection Committee, 71(13.65%) were online selected, and the remaining 137(26.35%) were selected through National Testing Service of Pakistan.

The article "Leadership empowering behaviour as a predictor of employees’ psychological well-being: Evidence from a cross-sectional study among secondary school teachers in Kohat Division, Pakistan" was retracted in 2025. Reasons: lack of ethics approval or compliance; missing or withdrawn patient consent; concerns about the welfare of human subjects.

**Table 3:** Participants’ demographic characteristics.

Characteristics	Categories	Frequency (*n*)	Percentage (%)
Gender	Male	353	67.88
	Female	167	32.12
Marital Status	Single	77	14.81
	Married	443	85.19
Age (in years)	25–30	64	12.31
	31–35	128	24.62
	36–40	113	21.73
	41–45	132	25.38
	46 and above	83	15.96
Teaching Experience (in years)	01–04	119	22.88
	05–09	221	42.50
	10–14	113	21.73
	15 and above	67	12.88
Nature of the Job	Permanent/Regular	520	100.0
	Adhoc	00	00.00
	Contract	00	00.00
Mode of Appointment	KPPSC	141	27.12
	DPC	171	32.88
	Online Selected	71	13.65
	NTS	137	26.35
Income Level	Rs. 30000 ≤ Rs. 39000	86	16.54
	Rs. 40000 ≤ Rs. 49000	165	31.73
	Rs. 50000 ≤ Rs. 59000	150	28.85
	Rs. 60000 & Above	119	22.88
Academic Qualification	Bachelor of Arts	56	10.77
	Master of Arts	449	86.35
	Master of Philosophy	12	02.31
	Doctor of Philosophy	03	00.58
Professional Qualification	Bachelor in Education	380	73.08
	Master in Education	128	24.62
	Master of Philosophy in Education	09	01.73
	Doctor of Philosophy in Education	02	00.38
Family Structure	Nuclear Family	169	32.50
	Joint Family	270	91.92
	Extended Family	81	15.58
Locality	Urban	193	37.12
	Rural	327	62.88

**Key:** KPPSC: Khyber Pakhtunkhwa Public Service Commission; DPC: Department Promotion Committee; NTS: National Testing Service.

The article "Leadership empowering behaviour as a predictor of employees’ psychological well-being: Evidence from a cross-sectional study among secondary school teachers in Kohat Division, Pakistan" was retracted in 2025. Reasons: lack of ethics approval or compliance; missing or withdrawn patient consent; concerns about the welfare of human subjects.

With respect to income level, 86(16.54%) participants’ income level was Rs. 30000 ≤ Rs. 39000, 165(31.73%) participants’ income level was Rs. 40000 ≤ Rs. 49000, 150(28.85%) participants earned Rs. 50000 ≤ Rs. 59000, and 119(22.88%) participants has the income level equal to Rs. 60000 & Above. Regarding academic qualification, 56(10.77%) participants were bachelor’s degree holders, 449 (86.35%) were master’s degree holders, 12(02.31%) M.Phil degree holders, and 03(00.58%) were Doctorate degree holders. In terms of professional qualification, 380(73.08%) participants were bachelor’s degree holders, 128(24.62%) were master’s degree holders, 09(01.73%) were M.Phil degree holders, and 02(00.38%) were a Doctorate degree holders. With regard to family structure, 169(32.50%) participants were residing in nuclear family, 270(91.92%) were living in joint family, and the remaining 81(15.58%) were living in extended family setup. With respect to the locality, 193(37.12%) of the participants belonged to urban localities while 327(62.88%) participants belonged to rural localities.

### Descriptive statistical analysis

#### Principals’ leadership empowering behavior

Table 4 summarizes the descriptive measurement of principals’ leadership empowering behaviour (LEB) which shows that principals were engaged in empowering behaviour at secondary level. The overall mean score of LEB was rated 5.70 with standard deviation and variance 0.304 and 0.093 respectively which clearly shows the positive response of the participants about the LEB of their principals. The most rated subdomains of LEB were coaching for innovative performance (*mean = 5*.*74*, σ *= 0*.*407*, σ^*2*^ *= 0*.*165; SEM = 0*.*018)* and accountability for outcomes (*mean = 5*.*73*, σ *= 0*.*441*, σ^*2*^ *= 0*.*195*, *SEM = 0*.*019)* followed by information sharing (*mean = 5*.*71*, σ *= 0*.*586*, σ^*2*^ *= 0*.*343*, *SEM = 0*.*026)*. The other subdomains of LEB were rated as delegation of authority (*mean = 5*.*68*, σ *= 0*.*481*, σ^*2*^ *= 0*.*231; SEM = 0*.*021)*, self-development (*mean = 5*.*67*, σ *= 0*.*563*, σ ^*2*^ *= 0*.*317; SEM = 0*.*025)*, and self-directed decision making *(mean = 5*.*66*, σ *= 0*.*513*, σ^*2*^ *= 0*.*264; SEM = 0*.*023)*. It clearly indicates that principals of educational institutions were engaged in empowering behaviours to encourage their subordinates for better psychological well-being and performance.

**Table 4:** Descriptive analysis of the principals’ leadership empowering behaviour.

Variables	n	Min	Max	Mean ± SD(σ)	Range	σ^*2*^	SEM	Skewness		Kurtosis	
								Statistic	SE	Statistic	SE
Overall Leadership Empowering Behaviour	520	4.76	6.65	5.70 ± 0.304	1.89	0.093	0.013	0.243	0.107	0.533	0.214
Delegation of Authority	520	3.33	6.67	5.68 ± 0.481	3.34	0.231	0.021	˗ 0.859	0.107	2.026	0.214
Accountability for Outcomes	520	4.33	7.00	5.73 ± 0.441	2.67	0.195	0.019	˗ 0.081	0.107	0.751	0.214
Self-Directed Decision Making	520	3.67	7.00	5.66 ± 0.513	3.33	0.264	0.023	˗ 0.718	0.107	1.398	0.214
Information Sharing	520	3.00	7.00	5.71 ± 0.586	4.00	0.343	0.026	˗ 0.601	0.107	0.753	0.214
Self-Development	520	3.67	7.00	5.67 ± 0.563	3.33	0.317	0.025	˗ 0.548	0.107	0.732	0.214
Coaching for Innovative Performance	520	4.00	6.67	5.74 ± 0.407	2.67	0.165	0.018	˗ 0.513	0.107	1.617	0.214

**Key:** n = sample size; SD(σ) = Standard Deviation; σ ^2^ = Variance; SEM = Standard Error Mean; SE = Standard Error.

The article "Leadership empowering behaviour as a predictor of employees’ psychological well-being: Evidence from a cross-sectional study among secondary school teachers in Kohat Division, Pakistan" was retracted in 2025. Reasons: lack of ethics approval or compliance; missing or withdrawn patient consent; concerns about the welfare of human subjects.

#### Secondary school teachers’ psychological well-being

Table 5 portrays that secondary school teachers were found psychologically healthier. The overall mean score of teachers’ psychological well-being was rated 4.78 with standard deviation and variance as 0.122 and 0.015 respectively which plainly reflects that secondary school teachers were psychologically better. With respect to subdomains of teachers’ psychological well-being, it was also found that secondary school teachers were psychologically healthier with respect to all subdomains i.e., autonomy (*mean = 4*.*78*, σ *= 0*.*364*, σ^*2*^ *= 0*.*132; SEM = 0*.*016)*, environmental mastery (*mean = 4*.*77*, σ *= 0*.*333*, σ^*2*^ *= 0*.*111; SEM = 0*.*015)*, personal growth (*mean = 4*.*78*, σ *= 0*.*362*, σ^*2*^ *= 0*.*131; SEM = 0*.*016)*, positive relations with others (*mean = 4*.*77*, σ *= 0*.*362*, σ^*2*^ *= 0*.*131; SEM = 0*.*016)*, purpose of life (*mean = 4*.*78*, σ *= 0*.*342*, σ^*2*^ *= 0*.*117; SEM = 0*.*015*), and self-acceptance (*mean = 4*.*77*, σ *= 0*.*399*, σ^*2*^ *= 0*.*122; SEM = 0*.*015)*. Conclusively, the results revealed that secondary school teachers were psychologically healthier in their workplace.

**Table 5:** Descriptive statistics of seondary school teachers’ psychological well-being.

Variables	n	Min	Max	Mean ± SD(σ)	Range	σ^*2*^	SEM	Skewness		Kurtosis	
								Statistic	SE	Statistic	SE
Overall Psychological Well-being	520	4.38	5.14	4.78 ± 0.122	0.76	0.015	0.005	0.086	0.107	– 0.019	0.214
Autonomy	520	3.57	5.71	4.78 ± 0.364	2.14	0.132	0.016	– 0.435	0.107	0.209	0.214
Environmental Mastery	520	3.71	5.71	4.77 ± 0.333	2.00	0.111	0.015	– 0.056	0.107	– 0.299	0.214
Personal Growth	520	3.43	5.86	4.78 ± 0.362	2.43	0.131	0.016	– 0.352	0.107	0.329	0.214
Positive Relations with Others	520	3.43	5.71	4.77 ± 0.362	2.28	0.131	0.016	– 0.412	0.107	0.505	0.214
Purpose of Life	520	3.57	5.57	4.78 ± 0.342	2.00	0.117	0.015	– 0.398	0.107	0.276	0.214
Self-Acceptance	520	3.71	5.71	4.77 ± 0.349	2.00	0.122	0.015	– 0.194	0.107	– 0.266	0.214

**Key:** n = sample size; SD (σ) = Standard Deviation; σ^2^ = Variance; SEM = Standard Error Mean.

The article "Leadership empowering behaviour as a predictor of employees’ psychological well-being: Evidence from a cross-sectional study among secondary school teachers in Kohat Division, Pakistan" was retracted in 2025. Reasons: lack of ethics approval or compliance; missing or withdrawn patient consent; concerns about the welfare of human subjects.

### Inferential statistical analysis and hypotheses testing

#### Pearson’s product-moment correlation

Hypothesis 1. *A Statistically significant relationship exists between leadership empowering behaviour and teachers’ psychological well-being at secondary level*.

In order to test the research hypothesis, Pearson’s product-moment correlation was applied between leadership empowering behaviour and teachers’ psychological well-being. Table 6 indicates a bivariate Pearson correlation and the value of *r* was calculated as 0.780 which clearly shows a significant (*p* < 0.01) positive relationship between leadership empowering behaviour and teachers’ psychological well-being. It demonstrates that the higher the leadership empowering behaviour then the higher will be the teachers’ psychological well-being and vice versa. The results have also been explained via scatterplot (see Fig 2). The Table 6 also portrays that a moderate positive correlation (0.40 ≤ r ≤ 0.69) was found between four subdimensions of leadership empowering behaviour and teachers’ psychological well-being i.e., delegation of authority (*r =* 0.573**), accountability for outcomes (*r =* 0.624**), information sharing (*r =* 0.406**), and coaching for innovative performance (*r =* 0.572**). On the other hand, a statistically weak positive correlation (0.01 ≤ r ≤ 0.39) was found between two subdimensions of leadership empowering behaviours and teachers’ psychological well-being i.e., self-directed decision making (*r =* 0.369**) and self-development (*r =* 0.377**). So, the hypothesis “a statistically significant relationship exists between leadership empowering behaviour and teachers’ psychological well-being at secondary level” was accepted. It clearly shows that the higher the leadership empowering behaviours then the higher will be teachers’ psychological well-being and vice versa. The outcomes have also been clarified via scatterplot (see Figs 3–8).

**Fig 2:** Pearson’s product-moment correlation between leadership empowering behaviour and teachers’ psychological well-being. The scatterplot undoubtedly demonstrates a significant positive relationship between overall leadership empowering behaviour and teachers’ psychological well-being at secondary level.

**Fig 3:** Pearson’s product-moment correlation between delegation of authority and teachers’ psychological well-being. The scatterplot plainly reflects the significant positive relationship between delegation of authority (subdomain of leadership empowering behaviour) and Teachers’ psychological well-being at secondary level.

The article "Leadership empowering behaviour as a predictor of employees’ psychological well-being: Evidence from a cross-sectional study among secondary school teachers in Kohat Division, Pakistan" was retracted in 2025. Reasons: lack of ethics approval or compliance; missing or withdrawn patient consent; concerns about the welfare of human subjects.

**Fig 4:** Pearson’s product-moment correlation between accountability for outcomes and teachers’ psychological well-being. The scatterplot clearly shows the significant positive relationship between accountability for outcomes (subdomain of leadership empowering behaviour) and teachers’ psychological well-being at secondary level.

**Fig 5:** Pearson’s product-moment correlation between self-directed decision making and teachers’ psychological well-being. The scatterplot plainly depicts the significant positive relationship between self-directed decision making (subdomain of leadership empowering behaviour) and teachers’ psychological well-being at secondary level.

**Fig 6:** Pearson’s product-moment correlation between information sharing and teachers’ psychological well-being. The scatterplot indicates the significant positive relationship between information sharing (subdomain of leadership empowering behaviour) and Teachers’ psychological well-being at secondary level.

**Fig 7:** Pearson’s product-moment correlation between self-development and teachers’ psychological well-being. The scatterplot clearly represents the significant positive relationship between self-development (subdomain of leadership empowering behaviour) and teachers’ psychological well-being at secondary level.

**Fig 8:** Pearson’s product-moment correlation between coaching for innovative performance and teachers’ psychological well-being. The scatterplot plainly indicates the significant positive relationship between coaching for innovative performance (subdomain of leadership empowering behaviour) and teachers’ psychological well-being at secondary level.

**Table 6:** Pearson’s product-moment correlation analysis between leadership empowering behaviour and teachers’ psychological well-being.

Variables	Mean	SD	1	2	3	4	5	6	7	8
1. Delegation of Authority	5.68	0.481	1.000							
2. Accountability for Outcomes	5.73	0.441	0.370**	1.000						
3. Self-Directed Decision Making	5.66	0.513	0.239**	0.242**	1.000					
4. Information Sharing	5.71	0.586	0.248**	0.326**	0.149**	1.000				
5. Self-Development	5.67	0.563	0.286**	0.218**	0.202**	0.155**	1.000			
6. Coaching for Innovative Performance	5.74	0.407	0.333**	0.389**	0.183**	0.179**	0.308**	1.000		
7. Leadership Empowering Behaviour	5.70	0.304	0.673**	0.669**	0.569**	0.517**	0.631**	0.625**	1.00	
8. Psychological Well-being	4.78	0.122	0.573**	0.624**	0.369**	0.406**	0.377**	0.572**	0.780**	1.000

** Correlation is significant at 0.01 level (2-tailed).

The article "Leadership empowering behaviour as a predictor of employees’ psychological well-being: Evidence from a cross-sectional study among secondary school teachers in Kohat Division, Pakistan" was retracted in 2025. Reasons: lack of ethics approval or compliance; missing or withdrawn patient consent; concerns about the welfare of human subjects.

**Correlation Strength:** 0.01≤ r≤0.39 = Weak Relationship; 0.40≤ r≤ 0.69 = Moderate Relationship; r≥0.70 = Strong Relationship.

#### Multiple linear regression analysis

Hypothesis 2. *Leadership empowering behaviour positively predicts teachers’ psychological well-being at secondary level*.

As presented in Table 7, the regression model is statistically significant on the ground that the value of ANOVA was calculated as 162.84 which shows that the result is significant (F-ratio = 162.840, R^2^ = 0.656, ΔR^2^ = 0.656, *p* < 0.05) statistically. Similarly, in each case, the calculated t-value is greater than the table t-value at 0.05 level of confidence. Additionally, the table reflects that the value of R square is 0.656 which demonstrates that 66% of the variance of teachers’ psychological well-being is accounted for input variables in this model. The regression analysis showed that all the subdimensions of leadership empowering behaviour were found the substantial predictors and have a substantial positive influence on teachers’ psychological well-being. Among these predictors, accountability for outcomes (*β = 0*.*312*, *B = 0*.*086*, *SE = 0*.*008*, *CI = 0*.*070–0*.*103*, *t-value = 10*.*27*, *p < 0*.*05*) was investigated the strongest predictor followed by coaching for innovative performance (*β = 0*.*280*, *B = 0*.*084*, *SE = 0*.*009*, *CI = 0*.*067–0*.*101*, *t-value = 9*.*498*, *p < 0*.*05*), delegation of authority (*β = 0*.*266*, *B = 0*.*067*, *SE = 0*.*007*, *CI = 0*.*053–0*.*082*, *t-value = 9*.*012*, *p < 0*.*05)*, information sharing (*β = 0*.*153*, *B = 0*.*032*, *SE = 0*.*006*, *CI = 0*.*020–0*.*043*, *t-value = 5*.*503*, *p < 0*.*05*), and self-directed decision making (*β = 0*.*137*, *B = 0*.*033*, *SE = 0*.*006*, *CI = 0*.*020–0*.*045*, *t-value = 5*.*022*, *p < 0*.*05*) respectively in defining employees’ psychological well-being positively. On the other hand, self-development (*β = 0*.*095*, *B = 0*.*020*, *SE = 0*.*006*, *CI = 0*.*009–0*.*032*, *t-value = 5*.*022*, *p < 0*.*05*) was found the weakest predictor of employees’ psychological well-being. It undoubtedly indicates that delegation of authority, self-directed decision making, accountability for outcomes, information sharing, self-development, and coaching for innovative performance are the substantial predictors that positively influence employees’ psychological well-being. Conclusively, the hypothesis was accepted.

**Table 7:** Multiple linear regression analysis indicating the role of principals’ leadership empowering behaviour in predicting teachers’ psychological well-being.

Teachers‘ Psychological Well-being (Dependent Variable)															
Model		Unstandardized Coefficients		Standardized Coefficients	*t*	*Sig*.	95% Confidence Interval for B		Collinearity Statistics		*R*^2^	ΔR^2^	*F*	*Sig*.	*Durbin-Watson*
		*B*	SE	*β*			Lower	Upper	Tolerance	VIF					
Independent Variables	**(Constant)**	2.935	0.060		48.551	0.000	2.816	3.054			0.656	0.656	162.840	0.000	1.798
	**DA**	0.067	0.007	0.266*	9.012	0.000	0.053	0.082	0.771	1.298					
	**AO**	0.086	0.008	0.312*	10.270	0.000	0.070	0.103	0.725	1.379					
	**SDM**	0.033	0.006	0.137*	5.022	0.000	0.020	0.045	0.898	1.114					
	**IS**	0.032	0.006	0.153*	5.503	0.000	0.020	0.043	0.870	1.150					
	**SDT**	0.020	0.006	0.095*	3.374	0.001	0.009	0.032	0.851	1.175					
	**CIP**	0.084	0.009	0.280*	9.498	0.000	0.067	0.101	0.771	1.297					

* Significant Predictors

**Key:** DA = Delegation of Authority; A = Accountability for Outcomes; SDM = Self-Directed Decision Making; IS = Information Sharing; SDT = Self-Development; CIP = Coaching for Innovative Performance.

The article "Leadership empowering behaviour as a predictor of employees’ psychological well-being: Evidence from a cross-sectional study among secondary school teachers in Kohat Division, Pakistan" was retracted in 2025. Reasons: lack of ethics approval or compliance; missing or withdrawn patient consent; concerns about the welfare of human subjects.

## Discussion

The study was aimed to examine the leadership empowering behaviour as a predictor of teachers’ psychological well-being at secondary level in Kohat Division, Pakistan. Unfortunately, research on the relationship between leadership empowering behaviour and employees’ psychological well-being has been ignored although, this area is very important to be considered as most of the researches have provided evidence that leadership empowering behaviour is positively affecting organizational outcomes [17, 45, 46, 48, 49, 53, 54, 57, 61, 62]. Similarly, employees’ psychological well-being also leads to positive outcomes, improved work performance, and higher organizational productivity [29, 68–71, 73]. Therefore, the researchers have made an attempt to examine the leadership empowering behaviour as a predictor of teachers’ psychological well-being. So, this study will bring definitely a constructive revolution in school leadership and organizational productivity through psychologically healthier teaching staff.

In hypothesis–I, we predicted that there would be a significant relationship between leadership empowering behaviour and teachers’ psychological well-being at secondary level. The findings of the study supported the hypothesis and found that there was a significant positive relationship between leadership empowering behaviour and teachers’ psychological well-being. Furthermore, the study also revealed that all the subdomains of leadership empowering behaviour were found positively correlated with teachers’ psychological well-being. In these subdomains, accountability for outcomes was found the most rated subdomains followed by delegation of authority, coaching for innovative performance, information sharing, self-development, and self-directed decision making respectively. This cross-sectional study provided evidence that leaders who are engaged in empowering behaviours have a positive influence on their subordinates’ psychological well-being. In such an environment, the employees feel satisfaction psychologically and physiologically which enables them to fulfill their responsibilities excellently. The results of this investigation confirmed the findings of Winston and Patterson [85] who concluded that leaders having empowering behaviour can implement the rules and regulations in organizations and empowered employees will assist in making a conducive working environment where employees’ well-being, prosperity, and better performance sustained. Likewise, as indicated by Culbertson, Fullagar, and Mills [86], leaders play a crucial role in promoting employees’ well-being and performance. Furthermore, they added that successful leaders delegate authority and engage employees. Their findings suggest that employees will shape inspirational mentalities when leaders exhibit concern about their feelings when delegating authority.

The article "Leadership empowering behaviour as a predictor of employees’ psychological well-being: Evidence from a cross-sectional study among secondary school teachers in Kohat Division, Pakistan" was retracted in 2025. Reasons: lack of ethics approval or compliance; missing or withdrawn patient consent; concerns about the welfare of human subjects.

The second objective of the study was to examine the leadership empowering behaviour as a predictor of teachers’ psychological well-being. So, in hypothesis–II, we predicted that leadership empowering behaviour would predict teachers’ psychological well-being at secondary level. The multiple linear regression modeling provided evidence that leadership empowering behaviour predicts teachers’ psychological well-being. All the domains of leadership empowering behaviour i.e., delegation of authority, accountability for outcomes, coaching for innovative performance, information sharing, self-development, and self-directed decision making were found significant predictors of employees’ psychological well-being. It plainly revealed that when leaders empower their subordinates, then the subordinates will be feeling satisfaction psychologically and thus they will be all the more ready to obey rules and strategies and perform excellently to produce high-quality work. These findings are consistent with the findings of Park et al. [4] who found that leadership empowering behaviour has a positive impact on employees’ psychological well-being. Laschinger, Wong, McMahon, and Kaufmann [87] expressed that employees having accessibility to resources and information, having support from companions and supervisors, and having the opportunity to learn and progress within the working environment are probably going to sense feelings of empowerment. In the same way, Mendes and Stander [51] asserted that leaders who capitalize in employees’ development, encourage accountability, and ensure participative decision-making then their subordinates would be more disposed to experience psychological empowerment within the organization. Bester, Stander, and van Zyle [46] concluded that accountability and self-directed decision-making affect employees’ participation substantially which implies that leaders who create feelings of independence and affecting the working environment (as experienced by the employees) will experience a significant level of participation from their subordinates. Tripathi and Bharadwaja [88] found that there was a strong indirect effect of empowering leadership on general mental health through psychological empowerment. The findings of this study revealed the effectiveness of empowering leadership in forecasting positive health outcomes.

The article "Leadership empowering behaviour as a predictor of employees’ psychological well-being: Evidence from a cross-sectional study among secondary school teachers in Kohat Division, Pakistan" was retracted in 2025. Reasons: lack of ethics approval or compliance; missing or withdrawn patient consent; concerns about the welfare of human subjects.

This study suggests some implications. As the study found that leadership empowering behaviour predicts employees’ psychological well-being and therefore, to create an empowering and conducive working environment, the leader must eliminate their traditional leadership style and adopt empowering behaviour to enhance the institutional productivity and employees’ psychological well-being as higher psychological well-being can enhance employees’ job performance [70]. Secondly, in underdeveloped countries such as Pakistan, education leaders are constantly challenged to enhance the working environment and provide unique incentives for employees’ satisfaction and happiness. Hence, it is imperative that these leaders not only understand but also admit the importance of empowering leadership and integrate the fundamental demands of employees into their organization and decision-making process. Thirdly, there is a need to focus on effective leadership style because leadership style is an important tool of management and if utilized appropriately then it may enhance positive relations with subordinates, ensure a favorable organizational climate, and enhance service performance [89]. Fourthly, the findings of this research are beneficial for policymakers, planners, curriculum developers, educationists, and the ministry of education to formulate effective and comprehensive strategies for improving employees’ psychological well-being as employees’ psychological well-being has a strong relationship with their performance [70]. Finally, educational institutions should adopt and focus on leadership empowering behaviour if they wish to retain their employees as well as to increase institutional efficiency.

This study has a few limitations. Firstly, the study has used only a quantitative research methodology. Therefore, a mixed-method research methodology might be utilized to explore the same issue in future exploration. Secondly, the study has used standardized tools for measuring teachers’ perceptions of their leader empowering behaviour and their own psychological well-being. So, there might be a slight contradiction in the results if the same problem may be explored via self-created instruments. Thirdly, the study is basically a cross-sectional survey i.e., correlational study which does not demonstrate the cause and effect. So, future research should be focused on longitudinal research design to test the cause and effect. Finally, this investigation was carried out in only five districts of Khyber Pakhtunkhwa. The outcomes may vary somewhat if the same research study may conduct in all regions of Khyber Pakhtunkhwa. Thus, the study in all districts with a bigger sample size will remove this shortcoming.

The article "Leadership empowering behaviour as a predictor of employees’ psychological well-being: Evidence from a cross-sectional study among secondary school teachers in Kohat Division, Pakistan" was retracted in 2025. Reasons: lack of ethics approval or compliance; missing or withdrawn patient consent; concerns about the welfare of human subjects.

## Conclusions

The study provided evidence that there is a significant positive relationship between leadership empowering behaviour and teachers’ psychological well-being. Leadership empowering behaviour predicts teachers’ psychological well-being. It shows that when leaders empower their subordinates, then the subordinates will be feeling satisfaction psychologically and thus they will be more enthusiastic to obey instructions, regulations, and procedures and tend to ensure high-quality work. Therefore, it is suggested that a leadership empowering behaviour approach should be adopted to enhance employees’ psychological well-being to upsurge organizational productivity and efficiency. Future focus on leadership empowering behaviour must take into consideration for promoting employees’ psychological well-being in order to improve institutional productivity.

## Supporting information

S1 Data Data set regarding leadership empowering behaviour. (XLSX)

S2 Data Data set regarding teachers’ psychological well-being. (XLSX)
